# Selecting Endophytes for Rhizome Production, Curcumin Content, Biocontrol Potential, and Antioxidant Activities of Turmeric (Curcuma longa)

**DOI:** 10.1155/2022/8321734

**Published:** 2022-08-23

**Authors:** Alain-Martial Sontsa-Donhoung, Marcelin Bahdjolbe, Hawaou, Dieudonné Nwaga

**Affiliations:** ^1^Soil Microbiology Laboratory, Biotechnology Centre, Faculty of Sciences, University of Yaoundé I, BP. 17673 Yaoundé, Cameroon; ^2^Department of Economic and Environmental Studies, National Education Centre, Ministry of Scientific Research and Innovation, BP. 6331 Yaoundé, Cameroon

## Abstract

Beneficial endophytes may enhance plant growth and stress tolerance. Yet, the plant health benefits of endophytes can be altered by biotic and abiotic factors and, thus, favour the inhibition of turmeric growth and curcumin production. The double petri dish method and greenhouse pot experiments were conducted to assess the biocontrol potential and impact of endophytes on the output, curcumin levels, and antioxidant activities of turmeric (*Curcuma longa* L.). The results showed that endophytes could control some disease-causing plant pathogens: 52% of all isolates have an antagonistic action against *Fusarium oxysporum*, 43% against *Pythium myriotylum*, 35% against *Phytophthora megakarya*, and 56% against *Ralstonia solanacearum in vitro*. Eight months after sowing, most endophyte isolates can increase the yield of turmeric rhizomes on a sterile substrate after inoculation, with yields ranging from 42 to 105% higher than the control and 3 to 50% higher than the urea treatment. In addition, 52% endophytes isolate significantly raised curcumin levels after 8 months of culture (from 2.1 to 3.1%) compared to control (1.7%) and urea treatment (1.8%). These endophytes promote an increase in the levels of reduced glutathione (22%), total thiols (26%), and carotenoids (91%) in turmeric. The study concludes that, in general, the endophytes-turmeric association can stimulate turmeric rhizome production, curcumin, and the antioxidant activities of the plant. They can also be used as biocontrol agents for plant pathogens.

## 1. Introduction

Turmeric (*Curcuma longa* L.) is a member of the Zingiberaceae family and is cultivated in tropical and subtropical regions throughout the world. It is native to India and Southeast Asia [1]. Turmeric powder is widely used as a colouring and flavouring agent in curries and mustards [2]. It has been traditionally used for medical purposes for many centuries in countries like India and China [3]. Turmeric is one of the most popular medicinal herbs, with a wide range of pharmacological activities. In general, turmeric has become an important source of new drugs for a variety of conditions, as the species contain molecules with validated antifungal, anti-inflammatory, hepatoprotective, antitumour, antiviral, and anticancer properties [4]. The pharmacological activity of turmeric has been attributed mainly to curcuminoids, composed of curcumin and two related compounds, demethoxycurcumin and bisdemethoxycurcumin [1]. Curcumin is the largest portion responsible for the biological activities of turmeric. Curcumin (diferuloylmethane), the major yellow bioactive component of turmeric, has been shown to have a broad spectrum of biological actions. These include anti-inflammatory, antioxidant, anticarcinogenic, antimutagenic, anticoagulant, antifertility, antidiabetic, antibacterial, antifungal, antiprotozoal, antiviral, antifibrotic, antivenom, antiulcer, hypertensive, and cholesterol-lowering activities. Its anticancer effect is mainly mediated by induction of apoptosis [5]. However, turmeric production presents many difficulties, and the production is limited in time. Turmeric is vulnerable to some air and soil-borne fungal diseases. The main symptoms on crops are rhizome rot (*Pythium aphanidermatum* and *Fusarium oxysporum)* and leaf spot (*Taphrina malucans*) [6].

These various biotic and abiotic stresses to which the plant is subjected contribute to the production of reactive oxygen species (ROS). Excess ROS is harmful to plants, as it can lead to lipid peroxidation, protein oxidation, DNA damage, and activation of programmed cell death [7]. Whether ROS play a harmful or signalling role depends on the production and elimination of ROS by the plant's defence system, which consists of antioxidant enzymes such as superoxide dismutase (SOD), catalase (CAT), glutathione peroxidase (GPX), and ascorbate peroxidase (APX) and nonenzymatic antioxidants such as ascorbic acid (ASA), tocopherols, and glutathione [8]. However, to our awareness, there is a lack of published data on the effect of endophytes in stimulating the production of rhizome, curcumin, and nonenzymatic antioxidant molecules from turmeric. The present study was conducted to assess the effect of endophytes on rhizome growth and production, stimulation of curcumin, reduced glutathione (GSH), total thiols (TT), and carotenoids contents of turmeric rhizomes on the one hand, and on the other hand, to evaluate the antimicrobial activities of endophytes.

## 2. Materials and Methods

### 2.1. Plant and Microbial Material

Turmeric rhizomes obtained from a previous turmeric crop in the greenhouse of the University of Yaounde I (Cameroon) were used as seeds to assess the effect of endophytes on turmeric. A total of 23 endophyte (20 bacterial: ClCaTb1, ClCaTb2, ClCaDj1, ClCeBe1, ClCeDs1, ClCeEb1, ClCeEb2, ClCeNk1, ClCeTb2, ClGlBe2, ClGlDj4, ClGlNk1, ClKbDs1, ClKbDs3, ClKbDl2, ClKbDl3, ClKbBi2, ClKbNk1, ClSgDj1, and ClSgNk3; and 3 fungal isolates: ClCeDs2, ClCeNk2, and ClPdBi1) isolated from the rhizosphere of turmeric, 2 bacterial isolates including 1 nitrogen-fixing bacteria (NFB) and 1 phosphorus solubilizing microorganism (PSM) from the bank of the Biotechnology Centre of the University of Yaoundé I, and 1 arbuscular mycorrhizal fungus (AMF) inoculum from the GIC Agribiocam were used as microbial material. The plant pathogens used for antimicrobial tests were *Fusarium oxysporum*, *Phytophthora megakarya*, *Pythium myriotylum*, and *Ralstonia solanacearum*.

### 2.2. Preparation of Microbial Inocula

For the preparation of bacterial inocula, 4-6 bacterial colonies were picked from the periphery of fresh isolates (24 hours). Each isolate was grown at room temperature under shaking in a 250 ml Erlenmeyer containing 100 ml of YMB liquid medium added to the peptone in the absence of light for 48 h. Inoculum concentration (1.7 × 10^8^ CFU/ml) was determined by colony counting [9]. For fungal inocula, mycelial pellets were collected from the periphery of 4–7-day old moulds on PDA (Potatoes Dextrose Agar). Isolates were grown for 7 days under natural diffuse light at 23-26°C on an agar nutrient medium; fungi were then covered with sterile distilled water for 3 days before being placed at 4°C for 1 h [10]. The number of zoospores (10^8^ spores/ml) was adjusted using colony counting [9].

### 2.3. Pot Experiment

An experiment was conducted for 8 months in the greenhouse of the University of Yaounde I, Yaounde, Cameroon. About 2 rhizomes of 3-5 knots, surface-sterilized [11], were planted 20 cm deep in a 5 kg pot with autoclaved (4 h at 121°C) substrates: a mixture of forest soil and sand in proportions of 3 : 1 [12]. The physicochemical characteristics of the soil were as follows: Sandy of 51%, clay of 29.5%, loam of 19.5%, CEC pH 7 of 15.36 meq/100 g, pH (H_2_O) of 4.5, organic C of 2.8%, organic matter of 4.8%, total *N* of 1 g/kg, available *P* of 8.66 mg/kg, the sum of bases of 6.62%, and C/N of 27. Pots were arranged in nonrandomized 1 × 28 × 16 blocks comprising a variety of turmeric, 1 control, 23 test microbial inocula, 3 positive control microbial inocula (PSM, NFB, and AMF), and 1 urea treatment (46% nitrogen) with 16 plants per treatment. Urea and Myco F were introduced at doses of 3 and 5 g/pocket, respectively. The different inocula were introduced at 15 ml/pocket. The doses were taken at six weeks (stage 2 to 3 leaves) and 14 weeks.

### 2.4. Agronomic Parameters and Sample Collection

Leaf area, number of leaves, and collar diameter were recorded for each treatment from 30 DAS (days after sowing) to 210 DAS every 3 weeks. At harvest (8 months after sowing), turmeric rhizome production was assessed.

### 2.5. Curcumin Determination

Turmeric (curcumin 95%) was obtained from Biotikon, Germany, and used to prepare the curcumin standard solution for UV visible spectroscopy. An amount of 20 mg was accurately weighed and transferred to a 100 ml volumetric flask. Then, 50 ml of methanol was added to obtain a concentration of 400 *μ*g/ml stock solution. From stock solution, 0.025, 0.05, 0.075, 0.1, 0.125, 0.15, 0.175, and 0.2 ml solutions were taken and diluted to 10 ml with methanol to obtain concentrations of 1, 2, 3, 4, 5, 6, and 7 *μ*g/ml, respectively [13]. The absorbance was measured at 424 nm. The curcumin calibration curve was then plotted with absorbance on the *y*-axis and curcumin concentration on the *x*-axis (Figure 1).

Fresh rhizomes harvested 8 months after sowing were cleaned, washed with deionised water, sliced, and dried at 80°C in a hot air oven for 48 h. Dried rhizomes were ground to powder by an electronic mill [14]. To prepare the test solutions for UV visible spectroscopy, 5 mg of turmeric powder was accurately weighed and transferred into a 50 mL volumetric flask. Methanol was added up to the mark, and the resulting solution was used for analysis after 3 days of maceration under shaking followed by filtration. The absorbance was measured at 424 nm. The amount of curcumin in each sample was determined by reference to the curcumin calibration curve (Figure 1).

### 2.6. Biocontrol Activities

All endophytic isolates were tested against three moulds: *Fusarium oxysporum*, *Pythium myriothylum*, and *Phytophthora megakarya* for fungistatic activity as described by Fokkema [15]. Twenty-four-hour cultures of separate isolates were spotted onto fungal test cultures prepared on CtMA medium (carrot 250 g/L; glucose 10 g/L; mannitol 1.5 g/L; agar 15 g/L; pH 6.8 ± 0.2). The plates were incubated at room temperature for 7 days, and the percentage of growth inhibition (PGI) was calculated using the formula [16]: PGI (%) = (*C* − *T*)/*C* × 100. All endophyte strains were also screened for antibacterial properties against *Ralstonia solanacearum*, as described by Grange and Devey [17] taken up by Chen et al. [18]. 10 ml of the *Ralstonia solanacearum* suspension (10^8^ CFU/ml) was added to the YGPA medium (yeast extract 5 g/L; glucose 10 g/L; peptone 5 g/L; agar 15 g/L; pH 7.2 ± 0.2), and the mixture was poured into Petri dishes. 10 *μ*l (10^6^ CFU/ml) of isolates was deposited on 9 mm sterile discs inside YGPA dishes containing *Ralstonia solanacearum*. The plates were incubated at 28°C for 3 days, and the diameter of the clear halo surrounding the filter was measured. The plates without antagonists were used as controls.

### 2.7. Nonenzymatic Antioxidant Assay

A spectrophotometric approach was used to evaluate nonenzymatic antioxidants. Reduced glutathione (GSH) was according to Ellman's method [19]. A methanolic extract of turmeric (1 ml) was homogenized in 2 ml of 5% (*w*/*v*) sulfosalicylic acid under cold conditions. The homogenate was shaken, and 100 *μ*l of supernatants was mixed with 1500 *μ*l of Ellman's reagent. After 1 hour, the absorbance was taken at 412 nm. The GSH level was expressed as mmol/g f.w: [GSH] = ΔDO/(*ε* × *L* × *m*). Total thiols (TT) were estimated as described by Sedlak and Lindsay [20]. Fresh powder (1 g) was homogenized in 0.02 M Tris-EDTA (pH 8.2), and the homogenates were centrifuged at 10000 g for 10 min at 4°C. Aliquots (2 ml) of the supernatants were mixed with 4 ml of 0.02 M Tris–EDTA buffer (pH 8.2) and 0.1 ml of 0.01 M DTNB. The colour was allowed to develop for 5 min. The absorbance was measured at 412 nm. TT were calculated using the molar extinction coefficient of 13.100 M^−1^ cm^−1^ [21]: *C*0 = *A*/*ɛ* × *D*). Carotenoids were estimated as described by Verma et al. [22]. The sample (0.5 g) was homogenized with 3 mL of cold acetone for 1 min and filtered, the operation was repeated until the acetone was no longer coloured, and then 10 mL of petroleum ether was introduced into a 500 mL separating funnel fitted with a Teflon tap, followed by acetone extracts. Afterward, 75 ml of distilled water was added slowly. The supernatant was washed 3-4 times with distilled water to remove the acetone. The petroleum ether phase was collected in a 25 mL volumetric flask. The volume was adjusted to the mark with light petroleum ether. The absorbance was read at 450 nm. The OD values must be between 0.2 and 0.8. The total carotenoid content is given by the following formula: Total carotenoids (mg/g) = *A*_450_ × *V* × 10^4^/*A*_1cm_^1%^ × *M*.

*A*_450_ is the absorbance à 450 nm; *V* is the volume (ml); *A*_1cm_^1%^ is the absorption coefficient of total carotenoids in petroleum ether (2500); *M* is the sample mass

### 2.8. Data Analysis

The data obtained was compiled in a database system using Microsoft Excel. Descriptive statistics were performed. Duncan's test was used to assess statistical differences using SPSS software. Variables with *p* < 0.05 were considered significant at the 95% confidence interval (CI).

## 3. Results and Discussion

### 3.1. Growth Parameters of Turmeric Plants

Vegetative growth (collar diameter, number of leaves, and leaf area) of turmeric was significantly (*p* < 0.05) influenced by the inoculation with most of the endophyte isolates, as shown in Figure 2. The general trend indicates that the collar diameter and leaf area of the plants increase at a faster rate until the 5^th^ month of growth and then decreased. This trend is consistent with Manohar et al. [23] on turmeric. The slow growth from the 6^th^ month of development can be attributed to the nutrient transport from the leaves to the rhizomes. In general, in all tuber crops, as the size of the underground storage member increases, there will be a gradual decrease in the growth of the aerial parts [24]. Although TClCeEb1 was not the only treatment that had a positive effect on the vegetative growth of turmeric, very few treatments had a negative effect on growth compared to the control. The better plant performance with the majority of endophyte isolates is probably due to the fact that they can promote plant growth and improve plant nutrition [25, 26]. Growth promotion by endophytes (Figure 3) may be a consequence of nitrogen fixation; production of phytohormones, biological control of plant pathogens through production of antimicrobial agents, production of siderophores; competition for nutrients and induction of host acquired resistance, or improvement of mineral bioavailability [25, 26]. These results (Figure 2) corroborate the report of several researchers which revealed that organic products and biofertilizers (arbuscular mycorrhizal fungus, endophytes) increased the vegetative growth and biomass production effectively [25, 27, 28].

### 3.2. Turmeric Rhizome Production and Curcumin Content

Significant differences were noticed in the yield and curcumin content of turmeric due to the application of various inocula (Figure 4). Turmeric rhizomes were harvested 8 months after sowing and, in general, all treatments had a favourable response to inoculated endophytes for rhizome mass increase, except TClCeTb2 and TClKbDs1 (Figure 4(a)). Among the treatments, it is clear that rhizome yields of TClPdBi1 (17.89 g/plant) and TClSgDj1 (17.66 g/plant) were the highest, followed by TClCeDs1 (17 g/plant) and TClCeBe1 (16.11 g/plant) without significant differences. Turmeric amended with these treatments remained green longer and had a larger leaf area (Figure 2(c)), which allowed a longer photosynthetic process to produce carbohydrates for vegetative growth and would have resulted in a higher turmeric rhizome yield. The use of chemical fertilisers such as NPK contributes to an increase in rhizome production yields (up to +80%) as described by previous studies [26, 29, 30]. While in this study, selected endophytes increase production yields up to +105%. In fact, Samanhudi et al. [31] showed that AMF increases the fresh weight of *Temulawak* rhizomes. Suryadevara and Ponmurugan [32] also reported a significant improvement in rhizome weight (60%) and soil microbial population after inoculation with a bacterial suspension of diazotrophs compared to the respective controls. Furthermore, Kumar et al. [33] inoculated *Azotobacter chroococcum* in the turmeric rhizome and observed increases in leaf number, shoot height, shoot biomass, and rhizome biomass. This may be explained by the fact that rhizospheric and endophytic species are directly or indirectly involved in growth promotion and plant disease management [30]. Regarding curcumin production, the results show that the curcumin content increased for most of the treatments that received the endophytes (Figure 4(b)). Among the treatments, TClCeNk1 (3.1%) increased the curcumin content of the rhizomes 2-fold compared to the control, followed by ClSgDj1 (2.4%) and ClPdBi1 (2.4%) isolates which were the highest. The NFB (2.6%) and PSM (2.4%) control also contributed to a significant increase in curcumin content in turmeric rhizomes compared to the control. Furthermore, among the inocula tests, 52% of the treatments favoured an increase in the curcumin content greater than the urea treatment, and 74% of the treatments favoured an increase in the curcumin content greater than the control. Previous studies showed that the use of chemical fertilisers slightly increases the curcumin content of rhizomes (up to +15%) [26, 29, 30]; whereas the selected endophytes in this study significantly increase the curcumin content (up to +82%). Indeed, Yamawaki et al. [14] show that AMF inoculation has beneficial effects on turmeric growth and curcumin production. The increase in curcumin synthesis and content might be due to the increase in the activity of key enzymes involved in curcumin biosynthesis like diketide-CoA synthase (DCS) and curcumin synthase (CURS) [34].

### 3.3. Biocontrol Properties

*In vitro* screens for antagonistic activity were conducted by cocultivating endophytes with 4 of the major plant pathogens affecting crops in Cameroon, 3 fungal (*Pythium myriotylum*, *Fusarium oxysporum*, and *Phytophthora megakarya*) and 1 bacteria (*Ralstonia Solanacearum)* pathogens. In these studies, a relevant fraction of the endophytic bacteria showed antagonistic effects (Figure 5). Out of the 23 endophyte isolates, 13 isolates showed antibacterial activity against *Ralstonia Solanacearum*; 10 isolates showed antifungal activity against *Pythium myriotylum*, 12 against *Fusarium oxysporum*, and 8 against *Phytophthora megakarya*. It was observed that the isolate, ClCaTb1 and ClKbNk1, had both antibacterial as well as antifungal properties. ClCeEb2 and ClCeEb1 isolates were the most efficient against *Ralstonia Solanacearum* at inhibiting diameters of 2.3 and 1.8 cm, respectively (Figure 5(a)). This result conforms to the results of Zhou et al. [35], where BJ-1 and BJ-31 isolates were found to be effective in controlling *Ralstonia Solanacearum* diseases on ginger. ClCeEb2 and ClCeTb2 isolates were more effective against *Pythium myriotylum* with inhibition percentages of 90 and 86%, respectively (Figure 5(b)). The present results support the Dinesh [36] report in 2015 according to which *Bacillus GRB35 amyloliquefaciens* isolate had 78.51% inhibition of *Pythium myriotylum* growth in ginger. Isolates ClGlNk1 and ClKbDl2 were more efficient against *Fusarium oxysporum* with 80 and 60% inhibition percentages, respectively (Figure 5(c)). Similar effects were reported by Miles et al. [37] who studied the biological control potential of 100 fungal endophytes associated with *Espeletia* sp. against common crop pathogens, including *Rhizoctonia solani*, *Botrytis cinerea*, *Fusarium oxysporum*, and *Phytophthora infestans*. Their results indicated that all endophytic strains were highly effective against many pathogens. *Phytophthora megakarya* is the most virulent species of *Phytophthora*, which is responsible for cocoa brown rot. Under heavy and frequent rainfall conditions in Cameroon, *Phytophthora megakarya* can cause yield losses of 50 to 70% or even 100% if no control measures are taken [38, 39]. In our study, only one of the endophytes tested *in vitro* against *Phytophthora megakarya* showed antagonism with an inhibition percentage greater than 50%. The isolates ClSgNk3, ClCaTb2, and ClKbDl3 gave the best percentages of inhibition with values of 55%, 41%, and 41%, respectively (Figure 5(d)). This work is comparable to that of Fadiji and Babalola [40]; Agnes et al. [41] showed that endophytes inhibit the growth of *Phytophthora palmivora* on the *in vitro* and *in vivo* cocoa plant. Thus, the results indicated that endophytes exhibit antimicrobial activities against these 4 plant pathogens. The endophytes showing antimicrobial activity could have the metabolite(s) with antibiotic properties. They could also produce hydrolytic enzymes like protease and chitinase, responsible for the degradation of the cell wall of the pathogen. Natural compounds synthesized by endophytic fungi have been reported as inhibitors of a wide variety of animal and plant pathogens [42]. Chen et al. [43] isolated *Bacillus* endophyte from peanut root and showed that it produced antimicrobial compounds with inhibitory effects against *Aspergillus flavus* and *Ralstonia solanacearum*. Indeed, endophytes can inhibit infection and pathogen proliferation in the host directly through antibiotic production, enzyme production, competition, and parasitism or indirectly by inducing host-intrinsic resistance responses [40].

### 3.4. Antioxidant Activities

The plant developed many strategies to scavenge the excessive reactive oxygen species (ROS) and prevent their accumulation. These strategies employ enzymatic antioxidants and nonenzymatic antioxidants [8]. Endophytes were extensively studied regarding this issue and were found to stimulate many mechanisms that help plants not only to survive but also to grow healthy under stress conditions [44]. This study evaluated the potential of endophytes to stimulate the production of reduced glutathione (GSH), total thiols (TT), and carotenoids in turmeric (*Curcuma longa*). GSH is one of the very most important antioxidants in the cell that play a key role in the protection of plants against the various form of biotic and abiotic stresses [45]. In our study, few endophyte isolates (22%) stimulated GSH production compared to the control. ClCeDs1, ClCeBe1, and ClCeDs2 isolates were the ones that, when applied to turmeric, favoured better stimulation of GSH production compared to controls with respective values of 15.27, 14.71, and 14.45 mmol/g (Figure 6(a)). Thiols are one of the crucial metabolites that act as detoxicants and antioxidants [46, 47]. The results showed (Figure 6(b)) that only 26% of endophyte isolates stimulated TT production compared to the control. ClCeBe1, ClCeTb2, and ClCeDs1 isolates inoculate into turmeric contributed to the best increases in TT contents with respective values of 75.67, 80.79, and 132.37 *μ*mol/g protein. The biological importance of the thiol compounds is linked to the activity of the sulfhydryl group involved in the antioxidant and detoxification reactions [46, 47]. A few recent studies have shown that the inoculation of microorganisms on different cultures allowed for a stimulation of GSH and thiol production [48–51]. The increased GSH levels in the inoculated plants under normal conditions could be related to the involvement of GSH in the redox homeostasis [52] that is probably managed by the endophytes. Vitamins are essential not only for humans but also for plants. In their review, Asensi-Fabado and Munne'-Bosch [53] reported that all the plant-derived vitamins have antioxidant activity. They are powerful antioxidants, play an important role in redox chemistry, and are cofactors as well [53]. Such as TT, GSH, and some low molecular weight compounds containing sulfhydryl groups, carotenoids (vitamin A precursor) are considered to be important nonenzymatic antioxidants [54]. In the present study (Figure 6(c)), almost all endophyte isolates (91%) contributed to the increase in carotenoid content of biofertilized turmeric plants. ClKbDl2 and ClCeBe1 isolates were found to multiply the highest amounts of carotenoids, including 6.1 and 5.99 mg/g of turmeric powder. Previous results have treated the benefits of inoculating plants with microorganisms, which led to increased levels of carotenoids [51, 55]. The increase in TT and carotenoid levels in response to endophytes could be related to their action on turmeric metabolism. An increase in GSH, TT, and carotenoids in the inoculated plant support the ability of endophytes to increase the biological and medicinal quality of turmeric.

## 4. Conclusion

The effectiveness of endophytes as biofertilisers is still little known in the tropics, particularly in Cameroon. They have the potential to improve growth, increase rhizome yield, curcumin, reduced glutathione, total thiols, and carotenoids in turmeric. However, further research should be carried out in the future to investigate the potential of the best endophytes (ClCeNK1, ClPdBi1, ClSgDj1, ClCaTb1, ClCeDs1, ClKbNk1, and ClCeBe1) in the study to control plant diseases and production of other crops besides turmeric under field conditions, but also to determine the mechanisms of action of the above during the production of curcumin, sulphur compounds, and carotenoids.

## Figures and Tables

**Figure 1:** Standard calibration curve for curcumin.

**Figure 2:** Comparing endophytes isolates on turmeric growth under sterilized pot conditions 90 and 210 days after sowing. (a) Collar diameter, (b) number of leaves, (c) leaf area. Control: no inoculation; AMF: arbuscular mycorrhizal fungi: PSM: phosphorus solubilizing microorganism; NFB: nitrogen-fixing bacteria. (a–d) correspond to abcd. Bars with the same alphabetical letter are not significantly different from each other at the 5% threshold according to Duncan's test.

**Figure 3:** Examples of the influence of some endophytes on turmeric growth 7 months after sowing. C: control; Urea: urea treatment; ClCeEb1, ClCeNk1, and ClCeEb2: bacteria isolates.

**Figure 4:** Effect of endophytes on (a) fresh rhizomes yield of turmeric harvested and (b) curcumin content of rhizomes 8 months after sowing (the bars with the same alphabetical letter are not significantly different from each other at the threshold of 5% according to the Duncan test).

**Figure 5:** Box plot of the effectiveness of endophytes against some plant pathogens in vitro. (a) *Ralstonia solanacearum*, (b) *Pythium myriotylum*, (c) *Fusarium oxysporum*, and (d) *Phytophtora megakarya*.

**Figure 6:** Effect of endophytes on the non-enzymatic antioxidant content of turmeric rhizomes after 8 months. (a) Reduced glutathione content. (b) Total thiol content. (c) Carotenoids content (the bars with the same alphabetical letter are not significantly different from each other at the threshold of 5% according to the Duncan test).

## Data Availability

Data used to support the findings of this study can be obtained upon request to the corresponding author.
